RETRACTED

# The Value of m5C-Related lncRNAs in the Prognostic Assessment and Immunotherapy of Stomach Adenocarcinoma

**DOI:** 10.1155/2022/2747799

**Published:** 2022-06-07

**Authors:** Chenxi He, Xinying Zhu, Fanting Kong, Xiaochong Zhang, Xiukun Chai, Chunyan Zou, Dongqiang Zhao

**Affiliations:** ^1^Department of Gastroenterology, The Second Hospital of Hebei Medical University, Shijiazhuang, 050000 Hebei Province, China; ^2^Department of Gastroenterology, Xingtai People's Hospital, Xingtai, 054000 Hebei Province, China; ^3^Department of Gastroenterology, The Third Hospital of Hebei Medical University, Shijiazhuang, 050000 Hebei Province, China

## Abstract

Long noncoding RNAs (lncRNAs) are closely associated with a variety of tumors, including stomach adenocarcinoma (STAD). However, the role of 5-methylcytosine- (m5C-) related lncRNAs in STAD is still uncertain. This study investigated the value of m5C-related lncRNAs in prognostic evaluation and immunotherapy of STAD. STAD transcriptome sequencing data were downloaded from The Cancer Genome Atlas (TCGA) database, and m5C-related lncRNAs were screened by Pearson correlation analysis. A prognostic m5C-related lncRNA signature (m5CRLSig) associated with STAD was established using univariate and multivariate Cox regression analysis. We constructed a prognostic risk model for STAD with six m5C-related lncRNAs. The receiver operating characteristic (ROC) curve was used to examine the predictive efficacy. Univariate and multifactorial Cox regression analysis and principal component analysis (PCA) validated m5CRLSig as an independent factor of STAD prognosis. The clinicopathological characteristics of the model showed higher risk scores for stages II-IV, grade 3, N1-3, and death status. The calibration curve of a nomogram revealed that the nomogram had an excellent predictive function for survival risk. Furthermore, the expression of six m5C-related lncRNAs in STAD and paracancerous tissues was detected by quantitative real-time PCR (qRT-PCR), which verified the feasibility of the m5CRLSig as a prognostic marker for STAD. m5C-related lncRNAs were linked to multiple immune-associated pathways, according to gene set enrichment analysis (GSEA). CIBERSORT analysis indicated that m5CRLSig was involved in immune cell infiltration. Risk score was associated with immune checkpoint gene expression, immune function scores, and chemotherapeutic drug sensitivity. Therefore, m5CRLSig can efficiently assess the prognosis of STAD patients and can be used as a biological marker for immunotherapy.

## 1. Introduction

Gastric cancer ranks fifth in cancer incidence and fourth in mortality, and with the number of new cases exceeding one million per year, the disease seriously affects human life and health [1, 2]. The most frequent gastric cancer is STAD, which originates from the glandular epithelium of the gastric mucosa. The pathogenesis of STAD is very insidious, and the early clinical symptoms are atypical. Most patients present local or distant metastases at the time of diagnosis and are already in the progressive stage of STAD, losing the opportunity for radical surgical treatment [3]. In addition, tumor recurrence after surgery is also one reason for the high mortality rate among patients with STAD. Despite the development and progress in neoadjuvant chemotherapy, targeted therapeutic, and immunotherapy, the treatment effectiveness and prognosis of STAD are still unsatisfactory [4]. Due to the limitations of STAD treatment options, further research is critical for the identification of innovative prognostic indicators and potential therapeutic targets for STAD.

RETRACTED

N6-Methyladenosine (m6A), N1-methyladenosine (m1A), m5C, N7-methylguanosine (m7G), and 5-hydroxymethylcytosine (hm5C) are common types of RNA methylation modifications [5]. RNA m5C methylation indicates that the fifth C position of RNA cytosine is modified by methylation, which is a major posttranscriptional modification of RNA [6]. RNA m5C methylation plays an essential role in the regulation of RNA translation, stability, exiting the nucleus, and other biological processes [7]. Neurovascular, cardiovascular, and autoimmune diseases are closely related to m5C methylation regulation [8–10]. Furthermore, abnormal m5C methylation is linked to the onset and progression of some cancers. Upregulation of the m5C methyltransferase NSUN2 has been shown to contribute to the malignant advancement of gastric cancer cells [11]. Bioinformatics studies illustrated that the levels of m5C genes correlated with the prognosis of patients with breast cancer and colon carcinoma [12, 13]. Currently, there is a lack of comprehensive understanding of the value of m5C-related lncRNAs in the prognostic assessment of STAD.

lncRNAs have multiple roles in regulating gene expression at the transcriptional and translational levels, and they have been reported to act as biomarkers for tumor diagnosis, metastasis, and immunotherapy [14]. A study showed that lncRNA ZNRD1-AS1 and its variants contribute more to the development of lung cancer from different approaches, including in vivo and epidemiological investigations [15]. Moreover, lncRNAs can regulate target genes by methylation and influence cancer progression. For example, the lncRNA UBA6-AS1 inhibits the decay of UBA6 mRNA by modifying the methylation status of m6A, thus suppressing ovarian cancer cell malignancy [16]. The m6A demethylase ALKBH5 mediates the modification of the methylation of the lncRNA KCNQ1OT1, thus upregulating the expression of the HOXA9 gene and promoting the development of laryngeal squamous cell carcinoma [17]. Nevertheless, previous studies have focused primarily on m6A methylation. m5C modifications have been confirmed to be widely present in a variety of RNAs. Abundant m5C methylation sites have been identified in ncRNAs by high-throughput techniques [18, 19]. This suggests that m5C modifications are also prevalent in ncRNAs. However, the function of m5C in lncRNAs has not been extensively studied. Therefore, an in-depth investigation of the link between m5C methylation and lncRNA is necessary to explore its potential biological functions.

RETRACTED

The tumor microenvironment (TME) is the local ecological environment on which tumor cells depend, and it includes immune cells, endothelial cells, microvasculature, and cytokines [20]. The interaction between the tumor and the immune cells undergoes a remodelling of the immune system, and eventually, tumor cells use a series of mechanisms to undergo immune escape or tumor dormancy. lncRNAs regulate differentiation, proliferation, secretion factors, and other biological processes of immune cells in the TME, which influence tumorigenesis and development [21]. For instance, in oral squamous cell carcinoma, the lncRNA CRNDE is upregulated, and its knockdown suppresses the production of T cell immunoglobulin, thus activating the antitumor effects of CD8+ T cells [22]. Zhang et al. [23] reported that the lncRNA GATA3-AS1 promotes immune evasion of breast cancer cells by mediating effector T cell trafficking, stabilising the PD-L1 protein, and degrading the GATA3 protein. Furthermore, lncRNAs also participate in the regulation of the TME in hepatocellular carcinoma and prostate cancer [24, 25]. However, the impact of m5C-related lncRNAs for TME and immunotherapy in STAD has not been reported.

The search for novel immunological markers to improve the prognosis of STAD patients is particularly essential. Our study integrated clinical data from TCGA database for STAD samples. We used bioinformatics and statistical analysis to screen and validate six m5C-related lncRNAs with prognostic value for STAD. The association of risk scores with immune cell infiltration, immune checkpoint genes, immune cell function score, and chemotherapeutic drug sensitivity was then further investigated. This study is aimed at developing accurate biological indicators for the prognostic assessment and precise treatment of STAD.

## 2. Materials and Methods

### 2.1. Data Acquisition

We downloaded the transcriptome sequencing data and clinical data of STAD from TCGA database official website (https://portal. http://gdc.cancer.gov). Clinical data included age, gender, stage, grade, TNM stages, and survival status. Data with complete clinical information were further sorted after data download. Ultimately, RNA sequencing data was obtained for 375 STAD samples and 32 normal samples. The lncRNA annotation information was downloaded from the GENCODE database (https://www.gencodegenes.org).

RETRACTED

### 2.2. Differential Expression and Interaction Identification of m5C Methylation-Regulated Genes

Thirteen m5C methylation-regulated genes have been described in the published study, namely, YBX1, ALYREF, DNMT1, NSUN4, TRDMT1, TET2, NSUN7, NSUN6, NSUN5, NSUN3, NSUN2, DNMT3A, and DNMT3B [26]. The expression matrix of the 13 m5C methylation-regulated genes was obtained from RNA-seq transcriptome data. The R software “limma” was utilized to evaluate discrepancies in m5C methylation-regulated genes. The screening criteria were |log_2_fold change| > 1 and a false discovery rate (FDR) < 0.05. The STRING database (https://www.string-db.org) was used to build a protein-protein interaction (PPI) network including the 13 m5C methylation-regulated genes, and the correlations were analyzed using the “corrplot” function in R software.

### 2.3. Acquisition of m5C-Related lncRNAs and Construction of a Prognostic Risk Model

The lncRNA profiles were obtained from the RNA-seq dataset. Subsequently, Pearson correlation analysis of m5C genes with the lncRNA expression matrix was performed to obtain m5C-related lncRNAs for STAD (|correlation coefficient| > 0.3, *p* < 0.001). The m5C-related lncRNA expression data were combined with clinical prognostic information from STAD patients. The “survival” and “survminer” packages in the R language were used to conduct the survival analysis. The m5C-related lncRNAs associated with prognostic significance were identified by univariate Cox regression and Kaplan–Meier analysis using *p* < 0.05 as the threshold. Next, they were included in multivariate Cox regression analysis to obtain regression coefficients for key lncRNAs and construct a multigene risk model. The coexpression network was visualized using Cytoscape software.

### 2.4. Evaluation of the Prognostic Model of m5C-Related lncRNAs

The ROC curve was used to examine the predictive efficacy of the model. The m5C-related lncRNA prognostic model was verified as an independent element of STAD prognosis using univariate and multivariate Cox regression analysis. PCA plots were generated using the R package scatterplot3D.

### 2.5. Construction of Nomogram and Enrichment Analysis

The R language “rms” package was adopted to create the prognostic nomogram model. We plotted calibration curves to evaluate the consistency of the nomogram model. GSEA software (GSEA_4.1.0) was used for the enrichment analysis of multiple genes in this study.

RETRACTED

### 2.6. Expression of m5C-Related lncRNAs in Tissues by qRT-PCR

We collected 20 matched STAD and paracancerous tissues from Xingtai People's Hospital. Pathologists histopathologically confirmed the diagnosis of all tissues. All patients had not received chemotherapy, radiotherapy, targeted drugs, immunotherapy, or Chinese herbal medicine. Patients were not diagnosed with malignancy at other sites or with other serious underlying diseases. The Ethics Committee of the Xingtai People's Hospital authorised this research. All patients signed the informed consent form before surgery. The specimens were removed and rapidly frozen in liquid nitrogen and stored in a low-temperature refrigerator at -80°C for subsequent studies. Then, the qRT-PCR experiment was carried out using the thermal cycler (Shanghai Qiqian Electronic Technology Co., Ltd., model: Q2000A). *β*-Actin was selected as the internal reference.

### 2.7. Immunocorrelation Analysis and Drug Sensitivity Analysis of Prognostic Features

We filtered with the Perl programming language to obtain the matrix of immune infiltrating cells and used CIBERSORT for immune infiltration analysis. Immunocorrelation analysis was visualized with the R packages “barplot,” “corrplot,” and “ggplot2.” Enrichment scoring of immune cells and immune function was performed by applying the single sample gene set enrichment analysis (ssGSEA). We compared the difference in the half inhibitory concentration (IC50) values of chemotherapeutic agents used for STAD treatment using “pRRophetic” in the R package.

### 2.8. Statistical Analysis

The R software (version 4.0.3) and the Perl software (version 5.3) were mainly applied for statistical analysis of the data. In this study, univariate and multifactorial Cox regression, Kaplan–Meier method, PCA, and ROC analysis were used. The Kruskal-Wallis test was used to compare differences between groups. The remaining analysis was performed as previously described. Two-tailed *p* < 0.05 was the threshold for statistical significance.

## 3. Results

### 3.1. Differential Expression and Interactions of m5C Methylation-Regulated Genes

The expression of 13 m5C methylation-regulated genes was analyzed in 375 STAD samples and 32 normal samples from TCGA database. The outcomes revealed that NSUN2, NSUN3, NSUN4, NSUN5, NSUN6, DNMT3A, DNMT3B, ALYREF, DNMT1, TRDMT1, and YBX1 were expressed at high levels in STAD samples (*p* < 0.05). Nevertheless, no significant differences were observed in the expression levels of NSUN7 and TET2 in the two types of samples (*p* > 0.05, Figure 1(a)). We constructed a PPI network of m5C methylation-regulated genes in STAD. Except for YBX1, there was a close interrelationship between the regulatory genes (Figure 1(b)). The node count showed that TRDMT1 interacted with the other seven m5C methylation-regulated genes and was a key factor in the relationship network (Figure 1(c)). DNMT3A and DNMT3B had the strongest connection, among the correlation analysis of 13 m5C methylation-regulated genes (Figure 1(d)). This indicates that the expression levels of m5C methylation-regulated genes in STAD samples and normal samples are different, and there is a certain interconnection between them.

RETRACTED

### 3.2. Identification of a Prognostic m5C-Related lncRNA Signature

Based on the data of STAD patients in TCGA database, we applied coexpression analysis to obtain 565 m5C-related lncRNAs. Univariate Cox regression and Kaplan–Meier analysis identified 10 m5C-related lncRNAs with prognostic value, which were AC009948.1, IPO5P1, AP001528.2, HAGLR, BOLA3-AS1, AC005586.1, SREBF2-AS1, AL590666.2, AP001271.1, and AL365181.3 (*p* < 0.05, Supplementary Table 1). Subsequently, the six prognostic m5C-related lncRNAs necessary to create the risk model were determined using multivariate Cox regression analysis (*p* < 0.05, Table 1). The correlations of these six lncRNAs with the m5C genes are presented in Figures 2(a) and 2(b). Of these, AC005586.1, AL590666.2, AP001271.1, and IPO5P1 were considered protective effectors (HR < 1, *p* < 0.05). HAGLR and AC009948.1 were considered risk effectors (HR > 1, *p* < 0.05). The expression correlations of m5C genes and m5C-related lncRNAs were compared in this study, and they were all positively correlated (*p* < 0.05, Figure 2(c), Supplementary Figure 1). Among them, DNMT3A and IPO5P1 correlated the strongest (Cor = 0.44, *p* = 1.073*e* − 20).

The risk score for STAD patients was calculated on the basis of the following formula. Risk score = (EXP HAGLR × 0.139064203280377) + (EXP AC009948.1 × 0.184190132013409) + (EXP AC005586.1×−0.21462505604275) + (EXP AL590666.2×−0.0333743988485729) + (EXP AP001271.1×−0.29068225147328) + (EXP IPO5P1×−0.286485959190337). EXP indicates the expression level of m5C-related lncRNAs. Patients with STAD were divided into high- and low-risk groups according to the median risk score. The Kaplan–Meier survival curves revealed that overall survival (OS) was markedly shorter in the high-risk group (*p* < 0.001, Figure 3(a)). Patients in the high-risk group had a worse survival status, according to the risk curves and the survival status scatter plots (Figures 3(b) and 3(c)). The ROC curves were then used to assess the predictor capacity of this risk model for 1-, 2-, and 3-year OS of STAD patients. The areas under the curve (AUC) were 0.728, 0.704, and 0.730, respectively (Figure 3(d)). This implies that the use of m5CRLSig to predict the prognosis of STAD has a certain accuracy.

RETRACTED

### 3.3. m5CRLSig as an Independent Prognostic Factor for STAD

To explore whether m5CRLSig is an independent predictive factor for OS in STAD patients, we conducted univariate and multivariate Cox regression analyses (HR: 1.466, 95% CI: 1.312–1.637, *p* < 0.001, Figure 4(a); HR: 1.380, 95% CI: 1.230–1.547, *p* < 0.001, Figure 4(b)). The risk score remained an independent risk factor for prognosis in STAD patients after excluding clinical confounders. Time-dependent ROC curves were also used to examine the accuracy of model prediction at 1, 3, and 5 years, with AUC values of 0.728, 0.676, and 0.741, respectively (Figure 4(c)). The accuracy of risk score was considerably higher than other clinicopathological factors. Next, we performed PCA for STAD patients according to the genome-wide (Figure 4(d)), m5C genes (Figure 4(e)), m5C-related lncRNAs (Figure 4(f)), and six prognostic m5C-related lncRNAs (Figure 4(g)). PCA according to the first three methods was ineffective in distinguishing high- and low-risk groups. However, the PCA could clearly separate the two groups of patients according to six prognostic m5C-related lncRNAs. These results demonstrate that m5CRLSig is an independent predictor of the prognosis in STAD.

### 3.4. Correlation of m5CRLSig with the Clinicopathological Characteristics of Patients

We examined the impact of six m5C-related lncRNAs' expression levels on OS in STAD patients. Based on the expression levels of lncRNAs, we divided STAD patients into high- and low-expression groups, as shown in Figure 5. The risk effector HAGLR and AC009948.1 high expression groups had shorter OS (*p* < 0.05, Figures 5(a) and 5(b)). The protective effector AC005586.1, AL590666.2, AP001271.1, and IPO5P1 high-expression groups had longer OS (*p* < 0.05, Figures 5(c)–5(f)).

We investigated the relationships between the risk score and clinicopathological characteristics and evaluated whether m5CRLSig influenced STAD development. Risk scores were significantly correlated with stage, grade, N stage, and survival status (*p* < 0.05, Figure 6(a)). Further studies determined that stages II-IV, N1-3, and grade 3 had higher risk scores (*p* < 0.05, Figures 6(b)–6(d)). Patients with high-risk scores had a worse survival status (*p* < 0.001, Figure 6(e)). This implied that patients having high-risk scores were predisposed to present with advanced clinicopathological characteristics.

RETRACTED

### 3.5. Clinical Prognostic Nomogram

To predict the survival risk for patients with STAD, a clinical prognostic nomogram was also designed (Figure 7(a)). We plotted the calibration curves to estimate the agreement with the model predictions and the actual observations (Figure 7(b)). The results displayed that the calibration curve was close to the diagonal, indicating a favourable agreement between the projected and real observed values. Thus, the nomogram designed using m5CRLSig has an excellent predictive capacity for the prognosis of STAD patients.

### 3.6. Expression of m5C-Related lncRNAs in Tissues by qRT-PCR

The information from TCGA database revealed that AC005586.1, AL590666.2, AP001271.1, and IPO5P1 had low expression, while HAGLR and AC009948.1 were highly expressed in STAD samples. To verify the feasibility of the prognostic model, we measured the expression of lncRNAs in STAD tissues and paired normal paracancerous tissues by qRT-PCR. The primers utilized are presented in Table 2. The expression levels of HAGLR and AC009948.1 were markedly elevated in STAD tissues compared to paracancerous tissues (*p* < 0.001). This indicates that HAGLR and AC009948.1 may be oncogenic factors in STAD. The expression of AC005586.1, AL590666.2, AP001271.1, and IPO5P1 was significantly reduced in STAD tissues (*p* < 0.01, Figure 8). We validated the reliability of m5C-related lncRNAs as prognostic markers for STAD using qRT-PCR experiments.

### 3.7. GSEA Situation

We then utilized functional enrichment analysis to probe potential signalling pathways of m5C-related lncRNAs. We visualized two groups of the top 5 signalling pathways based on GSEA software. Gene Ontology (GO) pathway analysis illustrated that immunoglobulin binding, extracellular matrix structural constituent conferring compression resistance, sialyltransferase activity, collagen trimer, and the collagen-containing extracellular matrix signalling pathway were enriched in the high-risk group. Acetyltransferase activity, endonuclease activity, lysine N-methyltransferase activity, catalytic activity acting on DNA, and DNA synthesis involved in DNA repair were enriched in the low-risk group (Figure 9(a)). Kyoto Encyclopedia of Genes and Genomes (KEGG) pathway analysis revealed that glycosphingolipid biosynthesis-ganglio series, hematopoietic cell lineage, cytokine–cytokine receptor interaction, asthma, and neuroactive ligand-receptor interaction signalling pathways were enriched in the high-risk group. The low-risk group had higher levels of RNA degradation, glycosylphosphatidylinositol (GPI) anchor production, cell cycle, base excision repair, and homologous recombination (Figure 9(b)). This implies that m5CRLSig may influence STAD development through immune-related pathways.

RETRACTED

### 3.8. Correlation between m5CRLSig and Immune Cell Infiltration

To investigate the value of m5CRLSig in the TME, we analyzed 22 tumor immune cells using CIBERSORT and the output was visualized with a heatmap (Figure 10(a)). The violin plot illustrated that immune cell infiltration differed in the two groups (Figure 10(b)). Patients with STAD in the high-risk group had a higher infiltration abundance of NK cells activated, dendritic cells resting, and mast cells resting (*p* < 0.05). Conversely, the infiltration abundance of NK cells resting was decreased in the high-risk group (*p* < 0.05). This evidences that immune cell infiltration in STAD patients was involved in tumor risk stratification. This study described the relationship between the risk score and the immune cells. The risk score was positively associated with the level of NK cells activated (*R* = 0.16, *p* < 0.05), dendritic cells resting (*R* = 0.26, *p* < 0.001), and mast cells resting infiltration (*R* = 0.18, *p* < 0.05, Figure 10(c)). The above three types of immune cells may be linked to the poor prognosis. Furthermore, we presented the proportions of 22 immune cell infiltration in STAD patients and visualized the results with a barplot (Supplementary Figure 2). m5CRLSig can distinguish immune cells in STAD with diverse features. We then evaluated the role of m5CRLSig in enrichment scoring of immune cells and immune function by ssGSEA. The results revealed that the enrichment scores of multiple immune cell (aDCs, B cells, DCs, iDCs, macrophages, mast cells, neutrophils, pDCs, T helper cells, TIL, and Treg) were elevated in the high-risk group (*p* < 0.05, Figure 10(d)). Furthermore, immune function scores such as APC costimulation, CCR, HLA, parainflammation, T cell costimulation, type I IFN response, and type II IFN response were also significantly elevated in the high-risk group (*p* < 0.05, Figure 10(e)). These results imply that m5C-related lncRNAs are involved in the regulation of immune cell function.

### 3.9. The Value of m5CRLSig in Immunotherapy and Chemotherapy

Immune checkpoint inhibitors (ICI) act on immune checkpoints to enhance the immune response or relieve immune suppression. To evaluate the connection between the risk score and ICI, we examined the expression of immune checkpoint genes in the two groups (Figure 11(a)). The results displayed that 18 immune checkpoint genes (CD40, CD200R1, TNFSF4, TNFRSF8, CD48, LAIR1, CD86, NRP1, PDCD1LG2, CD28, TNFRSF4, BTLA, TNFSF18, CD200, CD27, CD40LG, TNFSF14, and HAVCR2) were more expressed in the high-risk group (*p* < 0.05). However, two immune checkpoint genes, TNFRSF14 and TNFRSF25, were expressed at higher levels in the low-risk group (*p* < 0.05). The findings suggest that m5CRLSig may be a predictor of ICI treatment. We applied risk scores to assess the sensitivity of STAD patients to commonly used chemotherapeutic agents. Patients with low-risk scores were significantly more sensitive to cisplatin and paclitaxel (*p* < 0.05, Figures 11(b) and 11(c)). This implies that patients in the low-risk group would respond more effective to chemotherapy and would have a favourable prognosis.

RETRACTED

## 4. Discussion

Research on the pathogenesis of gastrointestinal tumors has made impressive achievements in recent years, and methods for effective prognostic assessment are being explored [27, 28]. Using bioinformatics research methods, we can analyze genes and their internal relations from the system level. In-depth mining of key regulatory molecules in STAD is important for finding effective and reliable therapeutic targets for STAD. The m5C modification of RNA has a wide range of functions, including cell signalling, tissue development and differentiation, and cancer regulation [29]. In the prognosis of many diseases, such as gastric cancer, lncRNAs play a key role [30]. However, the study of m5C methylation in lncRNAs is still in its infancy [31]. We used TCGA database to download details of transcriptome sequencing and clinical information from STAD patients to filter out m5C-related lncRNAs that are closely associated with patient prognosis. Combined with bioinformatics database resources, we constructed a prognostic risk model for m5C-related lncRNAs in STAD. To our knowledge, this is the first study on the feasibility and accuracy of m5CRLSig in STAD.

Methylation modifications and lncRNAs affect tumorigenesis and progression through a complex regulatory network. A study revealed that the m6A reader YTHDC1 blocked ubiquitination between lncRNA LSG1 and ESRP2 and inhibited the advancement of renal cell carcinoma [32]. By altering the stability of lncRNA ZFAS1, the m6A methyltransferase METTL3 influenced autophagy and the development of nasopharyngeal cancer cells [33]. Bioinformatics studies have also indicated the prognostic characteristics of m6A-related lncRNAs in gastric cancer [34, 35]. At present, the mechanism and function of m5C methylation modifications in lncRNAs remain to be elucidated. Yan et al. [36] demonstrated that NSUN2 methyltransferase catalyses m5C methylation of the lncRNA FOXC2-AS1 and inhibits FOXC2 mRNA degradation, thus promoting gastric cancer cell malignancy. Therefore, systematically establishing the molecular regulatory network of m5C-related lncRNAs in STAD is essential to uncover reliable therapeutic targets.

RETRACTED

We observed the expression of m5C methylation-regulated genes in STAD samples and normal control samples based on gene transcript data and understood their interactions in this investigation. Among the 13 m5C methylation-regulated genes, 11 had markedly elevated expression in STAD samples. It is indicated that m5C methylation-regulated genes may be associated with the pathogenesis of STAD. Through a comprehensive analysis, we detected m5CRLSig with important prognostic value. In addition, the risk score was discovered to be an independent risk factor for the prognosis of STAD patients. The qRT-PCR results further confirmed the reliability of m5CRLSig as a prognostic marker for STAD. Patients with high-risk scores were prone to develop advanced clinicopathological characteristics. These findings imply that six m5C-related lncRNAs may play a role in the progression and prognosis of STAD and had potential clinical value.

Among the six m5C-related lncRNAs obtained from the data analysis of this study, HAGLR and AC009948.1 were risk genes, while AC005586.1, AL590666.2, AP001271.1, and IPO5P1 were protected genes. We reviewed the research related to these six lncRNAs in tumors and especially in gastric cancer. HAGLR has been studied in tumors and has been found to act as a procarcinogenic factor in multiple tumors, including gastric cancer and breast cancer [37, 38]. Hu et al. [37] proved that HAGLR accelerated gastric cancer cell proliferation and promoted gastric cancer cell resistance to 5-Fu by regulating the miR-338-3p/lactate dehydrogenase-A (LDHA) axis. In triple-negative breast cancer, HAGLR was found to be closely associated with tumor growth, and HAGLR knockdown restrained the aggressive proliferation of breast cancer cells [38]. Further animal experiments also showed that upregulation of HAGLR significantly accelerated tumor growth [38]. Wei et al. [39] exhibited that AP001271.1 could be used as a ferroptosis-related lncRNA, and it constituted a model with three other lncRNAs to evaluate the prognosis of patients with gastric cancer, which is similar to our experimental results. IPO5P1 has not been reported in gastric cancer, but bioinformatics studies imply that IPO5P1 is a prognostic factor in bladder cancer and correlates with the effects of immunotherapy [40]. Currently, studies of AL590666.2, AC009948.1, and AC005586.1 in the tumor field have not been covered, which provide new molecular targets for relevant studies in the future.

The identification of tumor immune characteristics can be of great benefit for precise immunotherapy and vaccine development [41]. lncRNAs have an important role in immune recognition and immune evasion of tumor cells [42]. For instance, lncRNA HOTTIP maintains high levels of PD-L1 on the surface of neutrophils, inhibiting T cell proliferation through cumulative immune depletion, leading to tumor cell evasion of immune surveillance [43]. Furthermore, m5C methylation can also participate in the regulation of the TME. Gao et al. [44] revealed that patients with oral squamous cell carcinoma with high m5C methylation scores had lower immune activity and a poor prognosis. What roles do m5C-related lncRNAs play in the TME? In pancreatic ductal adenocarcinoma, m5C-related lncRNAs have been reported to induce polarisation or infiltration of M2 phenotype macrophages [26]. In this research, we investigated the relationship between m5C-related lncRNAs and tumor immune cell infiltration in STAD. We discovered that the risk score was positively associated with the level of NK cells activated, dendritic cells resting, and mast cells resting infiltration. The above three types of immune cells may be linked to a poor prognosis in STAD. However, the infiltration abundance of NK cells resting was decreased in the high-risk group. Dynamic interactions between m5CRLSig and the tumor immune microenvironment can produce different clinical outcomes. The regulatory function of m5C-related lncRNAs in STAD immune cell infiltration may be dual and may be significant players in the process of tumor immune escape or immune dormancy. The prognostic role of m5CRLSig in STAD is to a certain degree related to tumor immune cell infiltration.

RETRACTED

According to GO and KEGG enrichment analyses, m5C-related lncRNAs are linked to multiple immunological-associated pathways, such as immunoglobulin binding. This study also investigated the impact of m5CRLSig on the enrichment score of immune cells and immune function. The enrichment scores of multiple immune cell were higher in the high-risk group, such as aDCs, iDCs, and macrophages. Importantly, several immune function scores, such as CCR, HLA, and parainflammation, were also significantly higher in the high-risk group. The findings suggest that m5C-related lncRNAs participate in the adjustment of multiple immune cell functions. This may also be one reason for the discrepancy in the effectiveness of immunotherapy in patients with different risk scores. ICI can prevent cancer cells from undergoing immune escape and has become an important treatment for malignancies [45]. In this study, 18 immune checkpoint genes were highly expressed in the high-risk group of patients. m5CRLSig could provide some reference for ICI treatment in STAD patients. Next, we assessed the sensitivity of STAD patients to conventional chemotherapeutic drugs. Patients in the high-risk group were poorly sensitive to cisplatin and paclitaxel, which may also be a reason for the adverse prognosis in this group. These results suggest that m5CRLSig could be a potential predictive marker for immunotherapy and chemotherapy.

RETRACTED

This research has certain limitations. The model we created was not tested in additional datasets outside of TCGA. Most of the study population was Caucasian; thus, the results may not be universally applicable to all races. The mechanism of action of AL590666.2, AC009948.1, and AC005586.1 in tumors was unclear. The outcome of bioinformatics analysis still needs to be confirmed by a large amount of sequencing data and clinical trials.

## 5. Conclusions

Based on TCGA database, we selected six m5C-related lncRNAs that were highly related to the prognosis of STAD patients. Importantly, m5CRLSig participate in the modulation of tumor immune cell infiltration and are closely associated with both the expression of immune checkpoint genes and the sensitivity of chemotherapeutic agents. The present study provides new potential biological markers for immune treatment of STAD.

## Figures and Tables

**Figure 1:** Differential expression and interactions of m5C methylation-regulated genes. (a) Heatmap of m5C methylation-regulated gene expression in STAD samples versus normal samples. The horizontal coordinates represent samples, and the vertical coordinates stand for m5C methylation-regulated genes. (b) PPI network of m5C methylation-regulated genes. (c) Number of nodes of m5C methylation-regulated genes. (d) Correlation analysis of the 13 m5C methylation-regulated genes. ^∗∗^*p* < 0.01 and ^∗∗∗^*p* < 0.001.

**Figure 2:** Correlation between prognostic m5C-related lncRNAs and m5C genes. (a) Application of Cytoscape to visualize the coexpression network of m5C genes and m5C-related lncRNAs. (b) Sankey plots showing the association between m5C genes, m5C-related lncRNAs, and risk types. (c) The m5C-related lncRNAs were positively correlated with the m5C genes (*p* < 0.05).

**Figure 3:** The prognostic value of six m5C-related lncRNAs for STAD patients. (a) Kaplan–Meier survival curves for both groups of patients (*p* < 0.001). (b, c) Risk curves and survival status scatter plots of STAD patients. (d) ROC curves to assess the predictive efficacy of the risk model (AUC > 0.7).

**Figure 4:** Verifying the independence of m5CRLSig. (a) Univariate and (b) multivariate Cox regression analyses of the relationship between multiple clinical variables (including risk scores) and OS. (c) ROC curves for clinicopathological factors and risk scores at 1, 3, and 5 years. PCA of the (d) genome-wide, (e) m5C genes, (f) m5C-related lncRNAs, and (g) six prognostic m5C-related lncRNAs.

RETRACTED

**Figure 5:** Relationship between the expression levels of six m5C-related lncRNAs and OS in STAD patients. (a, b) Kaplan–Meier survival curves displaying shorter OS in patients in the HAGLR and AC009948.1 high-expression group (*p* < 0.05). (c–f) OS was longer in patients in the AC005586.1, AL590666.2, AP001271.1, and IPO5P1 high-expression groups (*p* < 0.05).

**Figure 6:** Relationship between risk score and clinicopathological characteristics. (a) Heatmap illustrating the clinicopathological characteristics and expression of six m5C-related lncRNAs in the high- and low-risk groups. Association of the risk score with the (b) stage, (c) lymph node metastasis status, (d) grade, and (e) survival status. ^∗^*p* < 0.05 and ^∗∗^*p* < 0.01.

**Figure 7:** Clinical nomogram. (a) Clinical prognostic nomogram predicting patient survival risk. (b) Calibration curves of the clinical prognosis nomogram.

**Figure 8:** The expression of six m5C-related lncRNAs in STAD tissues and paracancerous tissues was measured by qRT-PCR. ^∗∗^*p* < 0.01 and ^∗∗∗^*p* < 0.001.

**Figure 9:** GSEA situation. Top 5 (a) GO and (b) KEGG signalling pathways in the two groups.

**Figure 10:** m5CRLSig is related to immune cell infiltration. (a, b) Heatmap and violin map of immune cell infiltration. (c) Relevance of the risk score to three types of immune cells. Enrichment scores of (d) immune cells and (e) immune function.

**Figure 11:** Relevance of m5CRLSig to immunotherapy and chemotherapy. (a) Differences in the expression of immune checkpoint genes in the two groups. (b, c) Sensitivity of the two groups to cisplatin and paclitaxel. ^∗^*p* < 0.05, ^∗∗^*p* < 0.01, and ^∗∗∗^*p* < 0.001.

**Table 1:** Six prognostic m5C-related lncRNAs.

Gene ID	HR	HR.95L	HR.95H	*p* value
HAGLR	1.14919788	1.080942112	1.221763638	8.53*E* − 06
AC009948.1	1.202244387	0.997015744	1.449717894	0.03577198
AC005586.1	0.806843905	0.662135526	0.983178007	0.033321578
AL590666.2	0.967176382	0.94215051	0.992867004	0.012590168
AP001271.1	0.747753238	0.578011142	0.967342779	0.026918065
IPO5P1	0.750897622	0.594871707	0.94784679	0.015923186

**Table 2:** Primer information for qRT-PCR.

Primer	Sequence	Primer length	Tm	Product size
AC009948.1-F	CTTTTGGAACTTGATGGCACCTTA	24	59.72	236 bp
AC009948.1-R	CCTGGAAACTCTGCTCTGTAACT	23	59.99	
IPO5P1-F	TCCACAATGGTGTTGGAGGG	20	59.89	77 bp
IPO5P1-R	CTCAGGACCACGGACTCTCA	20	60.61	
HAGLR-F	CGCCCTTTCTGACCTGCTTA	20	60.04	284 bp
HAGLR-R	TGGCAGTCGTCTGGACATTC	20	60.04	
AC005586.1-F	CCACCTGCTGTAACTTCCTCTTTAG	25	61.08	90 bp
AC005586.1-R	CCTTTGCCACTCATTTTCTTTCTGC	25	61.53	
AL590666.2-F	GCTGGAACTTAACGCTGTCG	20	59.56	267 bp
AL590666.2-R	GAATTTTGGAGAGGAAGTGGAAGAC	25	59.82	
AP001271.1-F	GAAAGTAATGACGCTGGTGAGTATG	25	59.99	124 bp
AP001271.1-R	TCTGTGTTTAAGGTTTTGAGGAGCA	25	60.86	
*β*-Actin-F	GGCTGTATTCCCCTCCATCG	20	61.80	154 bp
*β*-Actin-R	CCAGTTGGTAACAATGCCATGT	22	61.10	

RETRACTED

## Data Availability

This study analyzed data from The Cancer Genome Atlas (TCGA) (https://http://portal.gdc.cancer.gov/). These data are free and publicly available.

## Supplementary Materials

Supplementary Materials Table 1: univariate Cox regression and Kaplan–Meier analysis of m5C-related lncRNAs in STAD. Supplementary Figure 1: correlation between prognostic m5C-related lncRNAs and m5C genes. Supplementary Figure 2: barplot of the proportion of immune cell infiltration in the high- and low-risk groups. The 22 immune cells were labelled with various colours in the legend.
